The article "Spiking Correlation Analysis of Synchronous Spikes Evoked by Acupuncture Mechanical Stimulus" was retracted in 2023. Reasons: plagiarism; overlap with other authors' work.

# Spiking Correlation Analysis of Synchronous Spikes Evoked by Acupuncture Mechanical Stimulus

**DOI:** 10.3389/fncom.2020.532193

**Published:** 2020-11-16

**Authors:** Qing Qin, Ya-Jiao Liu, Bo-Nan Shan, Yan-Qiu Che, Chun-Xiao Han, Ying-Mei Qin, Jiang Wang

**Affiliations:** ^1^Tianjin Key Laboratory of Information Sensing & Intelligent Control, School of Automation and Electrical Engineering, Tianjin University of Technology and Education, Tianjin, China; ^2^School of Electrical and Information Engineering, Tianjin University, Tianjin, China; ^3^China Academy of Electronics and Information Technology, Beijing, China

**Keywords:** population signals, spike correlation, synchrony, log-linear model, state-space model, bayesian theory, acupuncture

## Abstract

Acupuncturing the ST36 acupoint can evoke the response of the sensory nervous system, which is translated into output electrical signals in the spinal dorsal root. Neural response activities, especially synchronous spike events, evoked by different acupuncture manipulations have remarkable differences. In order to identify these network collaborative activities, we analyze the underlying spike correlation in the synchronous spike event. In this paper, we adopt a log-linear model to describe network response activities evoked by different acupuncture manipulations. Then the state-space model and Bayesian theory are used to estimate network spike correlations. Two sets of simulation data are used to test the effectiveness of the estimation algorithm and the model goodness-of-fit. In addition, simulation data are also used to analyze the relationship between spike correlations and synchronous spike events. Finally, we use this method to identify network spike correlations evoked by four different acupuncture manipulations. Results show that reinforcing manipulations (twirling reinforcing and lifting-thrusting reinforcing) can evoke the third-order spike correlation but reducing manipulations (twirling reducing and lifting-thrusting reducing) does not. This is the main reason why synchronous spikes evoked by reinforcing manipulations are more abundant than reducing manipulations.

## Introduction

Different acupuncturing manipulations can evoke different rapid and immediate concentrated effects in the corresponding target organ (Ezzo et al., 2000). The nature of the acupuncture effect depends on information regulation, in which neural information regulation plays an important role. And spike response activities are products of the neural regulation. In recent years, the analysis of response activities evoked by acupuncture has focused on the single neuron spike train and been largely confined to feature extraction, such as the spiking rate, the variation coefficient, the embedded dimension, the correlation dimension, and the complexity (Han et al., 2011; Men et al., 2012; Zhou et al., 2012). Ensemble spike activities are rarely investigated. In order to accurately quantify the acupuncture effect for different manipulations, we chose ensemble spike events as the research object in order to extract the network collaborative relationship.

The article "Spiking Correlation Analysis of Synchronous Spikes Evoked by Acupuncture Mechanical Stimulus" was retracted in 2023. Reasons: plagiarism; overlap with other authors' work.

With the rapid development of multi-electrode acquisition technology, more synchronous spikes have been detected in animal behavior and stimuli experiments (Gerstein and Clark, 1964; Meister et al., 1994; Gray et al., 1995; Brown et al., 2004; Segev et al., 2004; Blanche et al., 2005). A synchronous spike event is the important manifestation of the network collaborative activity (Hebb, 1949). In acupuncture experiments, some research has shown that reinforcing manipulations can evoke more response activities and encourage a higher spiking rate than reducing manipulations (Li, 2009). On this basis we instigated statistical analysis for ensemble spike events in 20 trials and found that the numbers of response spikes evoked by reinforcing manipulations were far higher than reducing manipulations, which mainly embodies synchronous spike activities.

In the earlier research, a study of the network collaborative relationship focused on the statistical analysis of ensemble spike trains. First, the cross-correlation method was used to obtain the stationary dependency in pairs of neurons (Perkel et al., 1967). Then Aertsen, Fujisawa et al. introduced the concept of the time-varying joint spiking rate of two neurons, which extended the pair-wise stationary dependency to the pair-wise dynamic dependency (Aertsen et al., 1989; Fujisawa et al., 2008). Still later, more methods, such as unitary event analysis (Grün et al., 2002a,b; Grün, 2009) and the CuBIC test method (Staude et al., 2010a,b) turned to the extraction of the high-order dynamic dependency based on ensemble spike trains.

In recent research, this model-based analysis has been extensively investigated. The generalized linear model is one of the most common models (Chornoboy et al., 1988; Brown et al., 1998; Truccolo et al., 2004), in which each spike train is modeled as a discrete point process based on all spike events and the time-varying spiking rate is modeled as a linear-non-linear cascade framework. In this cascade framework, spike-histories of other neurons are linearly superposed and then the spiking rate is obtained from the non-linear exponential transformation of the superposition result. Some methods also introduce input stimulus into the linear superposition (Kim et al., 2011). The generalized linear model is a probability statistical model, in which dynamic dependencies among neurons are directly modeled as linear coupling parameters of the spike-history (Truccolo et al., 2004; Okatan et al., 2005; Pillow et al., 2008). However, because ensemble spike trains are modeled on the assumption that spike events of each neuron are independent, these models cannot provide the time-varying joint spiking rate of neural ensemble or accurately describe dynamic synchronous spike activities.

The article "Spiking Correlation Analysis of Synchronous Spikes Evoked by Acupuncture Mechanical Stimulus" was retracted in 2023. Reasons: plagiarism; overlap with other authors' work.

In this paper, we model ensemble spike trains as multivariable Bernoulli events and adopt a log-linear model to directly describe dynamic joint spike activities. Pair-wise and high-order spike correlations are the model parameters, which describe the dependency among the neural ensemble. Unlike the cross-correlation analysis, the log-linear model simultaneously extracts all pair-wise spike correlations. This avoids the effect of other neurons. Meanwhile the log-linear model can extract high-order spike correlations avoiding the effect of lower-order spike correlations. Some studies have shown that high-order dependencies cannot be neglected in ensemble spike activities and a log-linear model containing only up to pair-wise interactions cannot account for stimulus encoding (Montani et al., 2009; Roudi et al., 2009; Ohiorhenuan et al., 2010; Santos et al., 2010; Yu et al., 2011). This method is used to ensemble spike trains evoked by different acupuncture manipulations. And the Akaike information criterion (AIC) is used to test the goodness-of-fit of the model and to judge the existence of high-order spike correlations. Based on the optimal model, ensemble spike correlations evoked by different acupuncture manipulations are estimated.

## Method

### Log-Linear Model

For the neural ensemble comprised of *N* neurons, taking time *t* for example, we define N-dimension binary variables $X^{t}=\left({X_{1}}^{t},{X_{2}}^{t},\ldots ,{X_{N}}^{t}\right)$ as the ensemble spike pattern. ${X_{i}}^{t}$ represents the spike state of the *i* neuron. When ${X_{i}}^{t}=1$, it indicates that the spike event occurs at time *t*. When ${X_{i}}^{t}=0$, it indicates that the spike event does not occur at time *t*. So, there are 2^*N*^ spike patterns for the neural ensemble. For a given spike pattern *x* = (*x*_1_, *x*_2_, …, *x*_*N*_) (*x*_*i*_ = 0 or 1), we define the joint probability function of its occurrence as *p*(*x*|θ_*t*_), which is determined by θ_*t*_ (ensemble spike correlations). θ_*t*_ reflects the dependency relationship of the neuron ensemble. The dimension of θ_*t*_ is 2^*N*^ − 1 because the sum of joint probabilities of all spike patterns is 1, namely ∑ *p*(*x*|θ_*t*_) = 1. The logarithm of the joint probability function is defined as a linear function (Amari et al., 2003; Gütig et al., 2003; Kass et al., 2011; Long and Carmena, 2011; Pillow et al., 2013) and the log-linear model is as follows:

(1) $$\begin{array}{r} \log\;p(x|\theta_{t})=\sum_{i}\theta_{i}^{t}x_{i}+\sum_{i<j}\theta_{ij}^{t}x_{i}x_{j}+\sum_{i<j<k}\theta_{ijk}^{t}x_{i}x_{j}x_{k}\cdots \\ +\;\theta_{1\cdots N}^{t}x_{1}\cdots x_{N}-\psi (\theta_{t}), \end{array}$$

where $\theta_{t}={\left(\theta_{1}^{t},\theta_{2}^{t},\ldots ,\theta_{12}^{t},\theta_{13}^{t},\ldots ,\theta_{1\cdots N}^{t}\right)}^{\prime }$ are ensemble spike correlations and compose the θ coordinate (Amari, 2001; Nakahara and Amari, 2002). The number of model parameters θ_*t*_ is $C_{N}^{1}+C_{N}^{2}+C_{N}^{3}+\cdots C_{N}^{N}=2^{N}-1$. Because of ∑ *p*(*x*|θ_*t*_) = 1, ψ(θ_*t*_) = −log*p*({0, …, 0}) is the log normalization parameter.

The article "Spiking Correlation Analysis of Synchronous Spikes Evoked by Acupuncture Mechanical Stimulus" was retracted in 2023. Reasons: plagiarism; overlap with other authors' work.

Besides, we define the expectation of the joint spike (the synchronous spike) at time *t* as follows:

(2) $$\begin{array}{l} \begin{array}{l} \eta_{i}^{t}=E\left[X_{i}^{t}\right]=1*p\left(X_{i}^{t}=1\right)\\ \;=p\left(\left\{x_{i}^{t}=1,0,\ldots ,0\right\}\right)+\underset{j\left(j\neq i\right)}{\sum }p\left(\left\{x_{i}^{t}=1,x_{j}^{t}=1,0,\ldots ,0\right\}\right)\\ \;+\underset{j<k\left(j\neq i,k\neq i\right)}{\sum }p\left(\left\{x_{i}^{t}=1,x_{j}^{t}=1,x_{k}^{t}=1,0,\ldots ,0\right\}\right)+\cdots \\ +p\left(\left\{1,\ldots ,1\right\}\right),\;i=1,\cdots \;,N\\ \eta_{ij}^{t}=E\left[X_{i}^{t}X_{j}^{t}\right]=1*p\left(X_{i}^{t}=1,X_{j}^{t}=1\right)\\ \;=p\left(\left\{x_{i}^{t}=1,x_{j}^{t}=1,0,\ldots ,0\right\}\right)\\ +\underset{k\left(k\neq i,k\neq j\right)}{\sum }p\left(\left\{x_{i}^{t}=1,x_{j}^{t}=1,x_{k}^{t}=1,0,\ldots ,0\right\}\right)\\ \;+\underset{k<l\left(k\neq i,k\neq j,l\neq i,l\neq j\right)}{\sum }\\ p\left(\left\{x_{i}^{t}=1,x_{j}^{t}=1,x_{k}^{t}=1,x_{l}^{t}=1,0,\ldots ,0\right\}\right)\\ +\cdots +p\left(\left\{1,\ldots ,1\right\}\right),\;i<j\\ \;\vdots \\ \eta_{1\cdots N}^{t}=E\left[X_{i}^{t}\cdots X_{N}^{t}\right]=1*p\left(X_{1}^{t}=1,X_{2}^{t}=1,\ldots ,X_{N}^{t}=1\right)\\ \;=p\left(\left\{1,\ldots ,1\right\}\right). \end{array} \end{array}$$

Expectations $\eta_{t}={\left(\eta_{1}^{t},\eta_{2}^{t},\ldots ,\eta_{12}^{t},\eta_{13}^{t},\ldots ,\eta_{1\cdots N}^{t}\right)}^{\prime }$ compose the η coordinate. In order to facilitate writing, Ω_*k*_ represents all possible combination forms of the k-order subset. Then for all subsets, we can get Ω_1_ = {1, 2, …, *N*}, Ω_2_ = {12, 13, …}, Ω_3_ = {123, 124, …},…,Ω_*N*_ = {123…*N*}. If *I* ∈ {Ω_1_, …, Ω_*N*_}, the corresponding model parameter and expectation parameter can be written as $\theta_{I}^{t}$ and $\eta_{I}^{t}$. Similarly, the joint spike event is substituted by *f*_*I*_(*x*):

(3) $$\begin{array}{l} \begin{array}{l} f_{i}\left(x\right)=x_{i},\;i=1,\cdots \;,N\\ f_{ij}\left(x\right)=x_{i}x_{j},\;i<j\\ \vdots \\ f_{1\cdots N}\left(x\right)=x_{1}\cdots x_{N}. \end{array} \end{array}$$

Equations (1, 2) are simplified as follows:

(4) $$\begin{array}{l} p\left(x|\theta_{t}\right)=exp\left[\sum_{I\in \left\{\Omega_{1},\ldots ,\Omega_{N}\right\}}\theta_{I}^{t}f_{I}\left(x\right)-\psi \left(\theta_{t}\right)\right], \end{array}$$

(5) $$\begin{array}{l} \eta_{I}^{t}=E\left[f_{I}\left(x\right)|\theta_{t}\right],I\in \left\{\Omega_{1},\ldots ,\Omega_{N}\right\}. \end{array}$$

Some research has shown that the θ coordinate and η coordinate are dually orthogonal coordinates and non-zero high-order spike correlations represent the excess and paucity of high-order synchronous spikes (Amari and Nagaoka, 2000; Amari, 2001, 2009; Nakahara and Amari, 2002). But it is worth noting that non-zero high-order spike correlations are not equal to the expectations of the corresponding order joint spikes. For a given r-order subset, {η_*I*_} (*I* ∈ {Ω_*r*_}) is the expectation of synchronous spikes. Equations (4, 5) show that {η_*I*_} (*I* ∈ {Ω_*r*_}) depends not only on r-order spike correlations {θ_*I*_} (*I* ∈ {Ω_*r*_}) but also on higher-order spike correlations {θ_*I*_} (*I* ∈ {Ω_*r*_, …, Ω_*N*_}, *r* ≤ *N*).

The article "Spiking Correlation Analysis of Synchronous Spikes Evoked by Acupuncture Mechanical Stimulus" was retracted in 2023. Reasons: plagiarism; overlap with other authors' work.

### State-Space Method for Estimating Spike Correlations

We chose ensemble spike events of *n* trials as the research object to make the result statistically significant. $X^{t,l}=\left({X_{1}}^{t,l},{X_{2}}^{t,l},\ldots ,{X_{N}}^{t,l}\right)$ is defined as the ensemble spike pattern in the *l*-th trial at time *t*, which is a sample for the joint probability function *p*(*x*|θ_*t*_). Based on experimental data of *n* trials, the effective estimate of ${\eta_{I}}^{t}$ is equal to the joint spiking rate:

(6) $$\begin{array}{l} y_{I}^{t}=\frac{1}{n}\overset{n}{\underset{l=1}{\sum }}f_{I}\left(X^{t,l}\right),\;I\in \left\{\Omega_{1},\ldots ,\Omega_{N}\right\}, \end{array}$$

where *I* ∈ {Ω_1_, …, Ω_*N*_}, $y_{t}={\left(y_{1}^{t},y_{2}^{t},\ldots ,y_{12}^{t},y_{13}^{t},\ldots ,y_{1\cdots N}^{t}\right)}^{\prime }$. For the observation interval [0, *T*], *y*_1:*T*_ = {*y*_1_, *y*_2_, …, *y*_*T*_} are efficient estimates of joint spiking expectations at each time. According to the Bernoulli experiment, *n* trials are independent of each other and we assume that spike patterns for all time are also independent of each other. Based on Equations (4, 6), we can get the conditional probability function for all ensemble spike events of *n* trials, which is given as:

(7) $$\begin{array}{l} p(y_{1\;:\;T}|\theta_{1\;:\;T})=\prod_{l=1}^{n}\prod_{t=1}^{T}\exp[\sum I\in \{\Omega_{1},\ldots ,\Omega_{N}\}\theta_{I}^{t}f_{I}(X^{t,l})-\psi (\theta_{t})]\\ \;=\prod_{t=1}^{T}\exp[n(\sum I\in \{\Omega_{1},\ldots ,\Omega_{N}\}\theta_{I}^{t}y_{I}^{t}-\psi (\theta_{t}))]\\ \;=\prod_{t=1}^{T}\exp[n({y^{\prime }}_{t}\theta_{t}-\psi (\theta_{t}))], \end{array}$$

where θ_1:*T*_ = {θ_1_, θ_2_, …θ_*T*_}.

The article "Spiking Correlation Analysis of Synchronous Spikes Evoked by Acupuncture Mechanical Stimulus" was retracted in 2023. Reasons: plagiarism; overlap with other authors' work.

In order to estimate dynamics spike correlations, we adopted the idea of the discrete state-space model. Here state variables are spike correlations, which are unknown. And observation variables are the ensemble spike events of *n* trials, which are observable and known. Equation (7) defines the conditional probability function for the observation process. For state variables, the iterative process is defined as a first-order autoregressive model, which is given as:

(8) $$\begin{array}{l} \theta_{t}=F\theta_{t-1}+\xi_{t}, \end{array}$$

where *t* = 2, …, *T*. *F* is the first-order autoregressive parameter. ξ_t_ obeys the normal distribution, in which the mean is the zero vector and the covariance matrix is *Q*. And the initial value of state variables also obeys the normal distribution θ_1_ ~ ν(μ, Σ). Here we assume that the parameter Σ is constant and *w* = [*F, Q*, μ] is the unknown parameter set of the state process.

According to Equation (8), we know (θ_t_−*Fθ*_t−1_) ~ ν(0, *Q*) and get the prior probability function of the state process *p*(θ_1:*T*_|*w*). Then the log-likelihood function of the ensemble spike events of *n* trials can be written as:

(9) $$\begin{array}{l} \begin{array}{l} l\left(w\right)=\log\int p\left(y_{1:T},\theta_{1:T}|w\right)d\theta_{1:T}\\ \;=\log\int p\left(y_{1:T}|\theta_{1:T}\right)p\left(\theta_{1:T}|w\right)d\theta_{1:T}. \end{array} \end{array}$$

The unknown parameter set *w* can be estimated by maximizing this log-likelihood function. Meanwhile according to the Bayesian theory, the posterior probability function can be written as

(10) $$\begin{array}{l} p\left(\theta_{1:T}|y_{1:T},w\right)=\frac{p\left(y_{1:T}|\theta_{1:T}\right)p\left(\theta_{1:T}|w\right)}{p\left(y_{1:T}|w\right)}. \end{array}$$

By maximizing the posterior probability function, the unknown state (spike correlations) can be estimated (Dempster et al., 1977; Akaike, 1980; Shumway and Stoffer, 1982; Smith and Brown, 2003; Smith et al., 2004; Pillow et al., 2013).

### Selection of the Log-Linear Model

For the neural ensemble comprised of *N* neurons, Equation (4) is a full model, which contains spike correlations of all orders. We can construct its hierarchical models, such as *E*_1_ ⊂ *E*_2_ ⊂ ⋯*E*_*N*_. *E*_*r*_ (*r* = 1, 2, …, *N*) a hierarchical log-linear model, in which spike correlations that are greater than the r-order are set to zero. If the model contains more high-order correlation terms, apparently it can better describe the joint probability of the ensemble spike pattern. However, for the estimation of spike correlations, more high-order correlation terms do not mean better. This is because when high-order synchronous spike activities do not exist in the neural ensemble, high-order correlation terms will lead to a large statistical fluctuation for the parameter estimation and estimates of low-order spike correlations would be inaccurate. This phenomenon is an over-fitting of the model, so it is necessary to remove non-existent high-order correlation terms.

The article "Spiking Correlation Analysis of Synchronous Spikes Evoked by Acupuncture Mechanical Stimulus" was retracted in 2023. Reasons: plagiarism; overlap with other authors' work.

This paper adopts the Akaike information criterion (AIC) (Akaike, 1980) to choose the optimal model. AIC is based on the concept of the information entropy, which is a balance between the model complexity and the model goodness-of-fit. When AIC for a given model is small, it means that the model provides a good description for experimental data with fewer parameters. According to the log-linear model, AIC is defined as,

(11) $$\begin{array}{l} \begin{array}{l} \text{AIC}=-2\log\int p\left(\theta_{1:T}|y_{1:T},w\right)d\theta_{1:T}+2k\\ \;=-2l\left(w\right)+2k, \end{array} \end{array}$$

where *k* is the number of parameters, which is equal to the sum of the numbers of *w* = [*F, Q*, μ] (Akaike, 1980; Kitagawa, 1987). For a given r-order hierarchical model, the number of spike correlation parameters $\theta_{t}={\left[{\theta_{1}}^{t},\ldots ,{\theta_{12}}^{t},\ldots ,{\theta_{1\cdots r}}^{t}\right]}^{\prime }$ is $d=\sum_{k=1}^{r}\left(\begin{array}{c} N\\ k \end{array}\right)$, so the total number of parameters is *k* = *d*^2^ + *d*(*d* + 1)/2 + *d*, in which three terms, respectively, represent the numbers of *F*, *Q*, and μ.

In addition, the Bayesian information criterion (BIC) (Schwarz, 1978; Rissanen, 2009) is another common information measure. Compared to AIC, BIC replaces the second term *k* with *k*log*n*. BIC is defined as,

(12) $$\begin{array}{l} \text{BIC}=-2l\left(w\right)+k\log n. \end{array}$$

### Selection of the State Model

Besides the selection of high-order correlation terms, we should choose the dynamic change pattern of the state process, which is determined by state parameters: *F* and *Q*in Equation (8). There are three dynamic change patterns: (I) *F* = *I* (identity matrix) and *Q* = 0; (II) *F* = *I* and *Q* is estimated by the state-space method; and (III) *F* and *Q* are both estimated by the state-space method. In case (I), spike correlations are stationary. In cases (II) and (III), spike correlations are non-stationary. Here we similarly use AIC to select the optimal dynamic change pattern.

The article "Spiking Correlation Analysis of Synchronous Spikes Evoked by Acupuncture Mechanical Stimulus" was retracted in 2023. Reasons: plagiarism; overlap with other authors' work.

## Result

### Simulation Data Analysis

In this section, we generate two sets of simulation data with known model parameters (spike correlations) to, respectively, test the effectiveness of the state-space method and information criterions (AIC and BIC). Meanwhile the relationship between spike correlations and synchronous spikes is discussed.

#### Testing the State-Space Estimation Method

The first-order and second-order spike correlations (dashed lines in Figures 1B,C) are used to simulate ensemble spike activities (Figure 1A), which contain two neurons (*N* = 2). Besides, we can obtain synchronous spikes of two neurons, which are shown as blue raster at the bottom of Figure 1C. At time *t* = 125*ms* (red dashed box), both θ_1_ and θ_2_ (the green dashed line and the pink dashed line) have a significant increase. At this moment, the blue raster (Figure 1C) are very dense because of the high spiking rates of the two neurons. At time *t* = 375*ms* (black dashed box), θ_12_ (blue dashed line) has a significant increase. Conversely, θ_1_ and θ_2_ reduce. At this moment, the blue raster (Figure 1C) are relatively dense because of the high second-order spike correlation.

**Figure 1:** Estimation of spike correlations for simulation data of two neurons. **(A)** Simulated ensemble spike activities. The number of neurons is *N* = 2 and the number of trials is *n* = 100. **(B)** First-order spike correlations: true values (dashed lines) and their estimates (solid lines). **(C)** Second-order spike correlations: true value (dashed line) and its estimate (solid line). Blue raster, at the bottom, represent the synchronous spikes of the two neurons.

Then the state-space method is used to simulation data (Figure 1A) and estimates of θ_1_, θ_2_, and θ_12_ are shown in Figures 1B,C (green, pink, and blue solid lines), in which three gray intervals are, respectively, their 95% credible intervals. Results show that all of the spike correlations (the first-order and the second-order) lay within 95% credible intervals of their estimates. The effectiveness of the state-space method has been validated.

#### Testing the Akaike and Bayesian Information Criterions

In order to test the effectiveness of the Akaike and Bayesian information criterions, the log-linear model with known spike correlations is used to simulate ensemble spike activities of three neurons (*N* = 3). There are non-stationary first-order, second-order, and third-order spike correlations in this model. And the number of trials is also *n* = 100. Then we can construct its hierarchical models *E*_*r*_ (*r* = 1, 2, 3). These three hierarchical models are employed to fit simulation data and corresponding model parameters (spike correlations) are estimated by the state-space method. Meanwhile in order to test the importance of the data sample size, we analyzed different sample sets: *n* = 3, 5, 10, 20, 50, 100. For different sample sizes, AICs and BICs of three hierarchical models can be calculated. Results are shown in Tables 1, 2. Minimum values of AICs and BICs for the three hierarchical models are marked in blue.

The article "Spiking Correlation Analysis of Synchronous Spikes Evoked by Acupuncture Mechanical Stimulus" was retracted in 2023. Reasons: plagiarism; overlap with other authors' work.

**Table 1:** AICs for different sample sizes of simulation data.

**Number of trials**	***r* = 1**	***r* = 2**	***r* = 3**
*n* = 3	1,207	1,197	1,213
*n* = 5	1,960	1,902	1,919
*n* = 10	3,782	3,647	3,663
*n* = 20	7,851	7,595	7,609
*n* = 50	19,259	18,592	18,585
*n* = 100	37,759	36,362	36,325

**Table 2:** BICs for different sample sizes of simulation data.

**Number of trials**	***r* = 1**	***r* = 2**	***r* = 3**
*n* = 3	1,199	1,172	1,182
*n* = 5	1,957	1,891	1,906
*n* = 10	3,784	3,655	3,673
*n* = 20	7,860	7,622	7,644
*n* = 50	19,276	18,644	18,652
*n* = 100	37,783	36,432	36,416

Table 1 shows that for small sample sizes (*n* = 3, 5, 10, 20), the second-order hierarchical model *E*_2_ is chosen, whose AICs is minimal. For large sample sizes (*n* = 50, 100), the third-order hierarchical model *E*_3_ with the minimal AICs is chosen. BIC has the same result in Table 2. Because neuronal spiking is a random event, the analysis of the synchronous spike and the spike correlation must be based on enough sample data. Results from one or two trials have statistical significance, which also cannot represent entire ensemble response activities. When the sample size is large enough, AIC and BIC both choose the full model *E*_3_ as the optimal model. The effectiveness of the two information criterions has been validated.

#### Relationship Between Spike Correlations and Synchronous Spikes

For the neural ensemble containing two neurons, synchronous spikes of the two neurons are represents by blue raster in Figure 1C. At time *t* = 375*ms*, second-order synchronous spikes occurred frequently with the increasing of the second-order spike correlation θ_12_ (blue line). In addition, at time *t* = 125*ms*, although the second-order spike correlation is fixed at zero, second-order synchronous spikes still have an obvious increase. It is because that two first-order spike correlations θ_1_ and θ_2_ both display an obvious increase (>-3) at this moment. When the first-order spike correlations are smaller than −3, they have little effect on the synchronous spike and will not be taken into account.

The article "Spiking Correlation Analysis of Synchronous Spikes Evoked by Acupuncture Mechanical Stimulus" was retracted in 2023. Reasons: plagiarism; overlap with other authors' work.

For the neural ensemble containing three neurons, estimates of spike correlations are, respectively, shown in Figures 2B–D based on ensemble spike activities (Figure 2A). In the bottom of each panel, synchronous spikes are shown as raster figures. Estimated curves and raster figures for the same order have the same color. Results show that second-order (low-order) synchronous spike events are not only related to corresponding order spike correlations but also the third-order (high-order) spike correlation. Specifically, in the interval [450*ms*, 500*ms*], synchronous spikes of neurons 1-2 (blue raster) do not increase but reduce with the increasing of θ_12_(blue solid line), compared with the interval [100*ms*, 150*ms*]. This is because of a smaller θ_123_ (gray dotted line) in the interval [450*ms*, 500*ms*]. In addition, although θ_23_ (red solid line) in the interval [100*ms*, 150*ms*] is much smaller than the interval [0*ms*, 50*ms*], red raster of neurons 2-3 in these two intervals show no significant difference. This is because θ_123_ (gray dotted line) in [100*ms*, 150*ms*] is much bigger. Meanwhile Figure 2D shows that the third-order (high-order) spike correlation θ_123_ represents the third-order (high-order) synchronous spike events.

**Figure 2:** Estimation of spike correlations for simulation data of three neurons. **(A)** Simulated ensemble spike activities. The number of neurons is *N* = 3 and the number of trials is *n* = 100. **(B)** First-order spike correlations: θ_1_, θ_2_, and θ_3_ (green, pink, and yellow solid lines). **(C)** Second-order spike correlations: θ_12_, θ_13_, and θ_23_ (blue, cyan, and red solid lines). **(D)** The third-order spike correlation: θ_123_ (gray solid line). Raster with different colors at the bottom show the timing of corresponding order synchronous spikes.

### Acupuncture Data Analysis

In the acupuncture experiment, healthy Sprague Dawley rats (weight: 180–200 g, age: 2–3) were selected as subjects. Before the experiment, all of the rats were fed for 7 days to adapt to the standard laboratory environment. In the process of the experiment, subjects were anesthetized deeply by 20% ethyl carbamate (1.5 g/kg) for preparation. We trimmed the hair between T8-L6 on both sides of the dorsal midline, cut the back skin along this midline, and removed the subcutaneous fascia. After that, the erector spinae, spinous process on both sides of centrum between T13-L5 was taken out to expose the spinal cord. To keep the spinal cord from drying out, paraffin oil at a temperature of 38°C was injected into stitched skin flaps. And then we used a hairspring tweezer to cut the spine dura mater with the help of the anatomical microscope. The dorsal roots separated from L3-L5 intervertebral foramen were snipped by eye scissors at the proximal part. Lastly, nerve filaments of the L4 dorsal root were placed on electrodes. And then, we used the BIOPAC-MP150 physiological recorder to record the spike activity of spinal dorsal root neurons evoked by acupuncture. We adopted four common manipulations in the clinical treatment: (I) twirling reinforcing, (II) lifting-thrusting reinforcing, (III) twirling reducing, and (IV) lifting-thrusting reducing. The stimulus frequency was 100 times/min and the stimulus duration was *T* = 2.5*s* (for specific experimental details refer to references Men et al., 2011 and Xue et al., 2013). We chose the spike trains of three neurons in 20 trials as the research object and created statistical analysis on the spike events. The numbers of spike events of single neurons evoked by four manipulations are shown in Table 3. Under the condition of reinforcing manipulations (I and II), the numbers of spikes of the three neurons are far more than those under the condition of reducing manipulations (III and IV). The last two rows marked in red are the number of supernumerary spikes of the three neurons evoked by manipulation I and II, respectively.

The article "Spiking Correlation Analysis of Synchronous Spikes Evoked by Acupuncture Mechanical Stimulus" was retracted in 2023. Reasons: plagiarism; overlap with other authors' work.

**Table 3:** Number of spike events of each neuron evoked by four manipulations in 20 trials.

**Manipulation**	**Neuron 1**	**Neuron 2**	**Neuron 3**
I	874	1,027	1,035
II	1042	824	851
III	653	659	592
IV	596	647	622
I-III	221	368	443
II-IV	446	177	229

The number of synchronous spike events evoked by the four manipulations are shown in the first four rows in Table 4. Numbers in the fifth row marked in red are the number of supernumerary synchronous spikes evoked by manipulation I compared to manipulation III. And numbers in the sixth row are the number of supernumerary synchronous spikes evoked by manipulation II compared to manipulation IV. According to Tables 3, 4, we find that reinforcing manipulations can evoke more response spikes than reducing manipulations, which mainly embody synchronous spike activities. In order to theoretically explain this phenomenon through the viewpoint of spike correlation, this paper introduces the log-linear model and the state-space estimation method into the analysis of acupuncture data.

**Table 4:** Number of synchronous spike events evoked by four manipulations in 20 trials.

**Manipulation**	**Neurons 1-2**	**Neurons 1-3**	**Neurons 2-3**	**Neurons 1-2-3**
I	190	176	261	129
II	109	111	223	85
III	67	33	69	25
IV	70	57	94	41
I-III	123	143	192	104
II-IV	39	54	129	44

#### Selection of the Log-Linear Model and the State Model

The first step is to choose the appropriate models for the acupuncture data. Here because acupuncture is a discrete stimulation, we assume that the first-order autoregressive parameter *F* in the state model is not equal to the identity matrix and is optimized by the estimation method. Ensemble spike activities with different sample sizes (*n* = 2, 5, 10, 15, 20) evoked by the four manipulations are used to fit three hierarchical models (*E*_1_, *E*_2_ and *E*_3_). And their corresponding AICs can be calculated and shown in Tables 5–8. For the given sample sizes, the minimum values of AICs are marked in blue. Results show that under the condition of reinforcing manipulations (I and II), when the sample size is large enough (*n* = 20), AIC chooses the full model *E*_3_ as the optimal model. Conversely, under the condition of reducing manipulations (III and IV), the hierarchical model *E*_2_ is selected. Therefore, we conclude that reinforcing manipulations can evoke the third-order spike correlation θ_123_ and reducing manipulations cannot. This is the main reason why more response spikes are evoked by the two reinforcing manipulations.

The article "Spiking Correlation Analysis of Synchronous Spikes Evoked by Acupuncture Mechanical Stimulus" was retracted in 2023. Reasons: plagiarism; overlap with other authors' work.

**Table 5:** AICs for different sample sizes of acupuncture data evoked by manipulation I.

**Number of trials**	***r* = 1**	***r* = 2**	***r* = 3**
*n* = 2	1,875	1,846	1,884
*n* = 5	4,564	4,371	4,398
*n* = 10	8,882	8,485	8,509
*n* = 15	13,152	12,558	12,560
*n* = 20	NaN	16,663	16,635

**Table 6:** AICs for different sample sizes of acupuncture data evoked by manipulation II.

**Number of trials**	***r* = 1**	***r* = 2**	***r* = 3**
*n* = 2	1,744	1,696	1,727
*n* = 5	4,311	4,099	4,130
*n* = 10	8,180	7,765	7,803
*n* = 15	12,298	11,664	11,695
*n* = 20	16,635	15,767	15,744

**Table 7:** AICs for different sample sizes of acupuncture data evoked by manipulation III.

**Number of trials**	***r* = 1**	***r* = 2**	***r* = 3**
*n* = 2	1,297	1,345	1,384
*n* = 5	3,083	3,106	3,139
*n* = 10	6,184	6,150	6,182
*n* = 15	9,103	9,016	9,042
*n* = 20	12,156	11,986	12,003

**Table 8:** AICs for different sample sizes of acupuncture data evoked by manipulation IV.

**Number of trials**	***r* = 1**	***r* = 2**	***r* = 3**
*n* = 2	1,301	1,342	1,385
*n* = 5	3,102	3,059	3,100
*n* = 10	5,965	5,871	5,896
*n* = 15	8,816	8,667	8,687
*n* = 20	11,794	11,546	11,562

In the selection of the log-linear model, the autoregressive parameter *F* is fixed at the identity matrix. AICs of four chosen models have been calculated and we show them in the first row of Table 9. Meanwhile we calculate AICs (the second row of Table 9) of the four chosen models under the condition of the optimized *F*. For the four manipulations, AICs in the second row are less than those in the first row. The efficacy of the assumption that the state parameter *F* is optimized has been validated.

The article "Spiking Correlation Analysis of Synchronous Spikes Evoked by Acupuncture Mechanical Stimulus" was retracted in 2023. Reasons: plagiarism; overlap with other authors' work.

**Table 9:** AICs of given hierarchical models of the four manipulations for different state processes.

**State parameter**	**I, *r* = 3**	**II, *r* = 3**	**III, *r* = 2**	**IV, *r* = 2**
*F* = *I*	16,771	15,859	12,091	11,632
Optimized *F*	16,635	15,744	11,986	11,546

#### Analysis of Acupuncture Reinforcing Manipulations

This section discusses the twirling reinforcing manipulation and its ensemble response activities (Figure 3A) are used to fit the full model *E*_3_. In Figure 3A, each twirling reinforcing stimulus can evoke a lot of spike activities and spike times show a single-peak distribution. Based on spike trains in 20 trials, joint (synchronous) spike events (colored raster in Figure 3) and their rates (Figure 3B) can be obtained. Then the state-space method is used to estimate spike correlations. Figure 3C shows that three first-order spike correlations are <0. Only θ_1_ and θ_2_ are significantly >-3 during each acupuncture stimulus. Therefore, except for the synchronous spikes of neurons 1-2, the first-order spike correlations are not the main considerations for synchronous spike events.

**Figure 3:** Estimation of spike correlations for acupuncture data evoked by twirling reinforcing. **(A)** Ensemble spike activities. The number of neurons is *N* = 3 and the number of trials is *n* = 20. **(B)** Rates of joint spike: η_12_, η_13_, η_23_, and η_123_. **(C)** First-order spike correlations: θ_1_, θ_2_, and θ_3_ (green, pink, and yellow solid lines). **(D)** Second-order spike correlations: θ_12_, θ_13_, and θ_23_ (blue, cyan, and red solid lines). **(E)** Third-order spike correlation: θ_123_ (gray solid line). Raster with different colors at the bottom show the timing of corresponding order synchronous spikes.

Figure 3D shows that second-order synchronous spike events are not only related to corresponding order spike correlations but also to the third-order spike correlation θ_123_. Take the third acupuncture stimuli for example ([1.1*s*, 1.7*s*]), θ_12_ is negative in the interval [1.2*s*, 1.4*s*]. But because θ_123_ is large enough during this time period, there are many synchronous spikes of neurons 1–2 (blue raster). In the interval [1.4*s*, 1.5*s*], θ_12_ gradually increases, but the number of blue raster has a dramatic decline because of a smaller θ_123_. For the rest of the time ([1.5*s*, 1.7*s*]), values of θ_12_ and θ_123_ are both large. However, in this time period, the current stimuli has stopped. Therefore, the three first-order spike correlations are very small and spike activities disappear gradually. For synchronous spikes of neurons 1–3 and neurons 2-3, θ_13_ and θ_23_ are both larger than θ_12_ during the interval [1.25*s*, 1.45*s*]. So synchronous spikes of neurons 1-2 rely more on θ_123_. Figure 3E shows that synchronous spikes of neurons 1-2-3 (gray raster) increase with the increasing of θ_123_ during each acupuncture stimulus. Therefore, the third-order spike correlation θ_123_ represents third-order synchronous spike events.

The article "Spiking Correlation Analysis of Synchronous Spikes Evoked by Acupuncture Mechanical Stimulus" was retracted in 2023. Reasons: plagiarism; overlap with other authors' work.

For the lifting-thrusting reinforcing manipulations, analysis results are shown in Figure 4. From Figure 4A, we find that spike times during each acupuncture stimulus show a multi-peak distribution. Therefore, analysis results are same as twirling reinforcing, except for the characteristic of volatility. In addition, during each acupuncture stimulus θ_23_ (Figure 4D, red solid line) is larger than θ_123_ (Figure 4D, gray dotted line) and the red raster become dense with the increasing of θ_23_. Therefore, the dependence of synchronous spikes of neurons 2-3 on θ_123_ is minimal. And Figure 4E shows that synchronous spikes of neurons 1-2-3 (gray raster) are the result of the interaction of second-order and third-order spike correlations.

**Figure 4:** Estimation of spike correlations for acupuncture data evoked by lifting-thrusting reinforcing. **(A)** Ensemble spike activities. The number of neurons is *N* = 3 and the number of trials is *n* = 20. **(B)** Rates of joint spike: η_12_, η_13_, η_23_, and η_123_. **(C)** First-order spike correlations: θ_1_, θ_2_, and θ_3_ (green, pink, and yellow solid lines). **(D)** Second-order spike correlations: θ_12_, θ_13_, and θ_23_ (blue, cyan, and red solid lines). **(E)** Third-order spike correlation: θ_123_ (gray solid line). Raster with different colors at the bottom show the timing of corresponding order synchronous spikes.

#### Analysis of Acupuncture Reducing Manipulations

This section discusses the twirling reducing manipulation and its ensemble response activities (Figure 5A) are used to fit the hierarchical model *E*_2_. Its analysis results are shown in Figure 5. From Figures 5A,B, we find that spike times during each acupuncture stimulus also show a single-peak distribution, but the number of response spikes are less than the twirling reinforcing. The main reason is that reducing manipulations cannot evoke the third-order spike correlation.

**Figure 5:** Estimation of spike correlations for acupuncture data evoked by twirling reducing. **(A)** Ensemble spike activities. The number of neurons is *N* = 3 and the number of trials is *n* = 20. **(B)** Rates of joint spike: η_12_, η_13_, η_23_, and η_123_. **(C)** First-order spike correlations: θ_1_, θ_2_, and θ_3_ (green, pink, and yellow solid lines). **(D)** Second-order spike correlations: θ_12_, θ_13_, and θ_23_ (blue, cyan, and red solid lines). Raster with different colors at the bottom show the timing of corresponding order synchronous spikes.

The article "Spiking Correlation Analysis of Synchronous Spikes Evoked by Acupuncture Mechanical Stimulus" was retracted in 2023. Reasons: plagiarism; overlap with other authors' work.

Figure 5C shows that, like the twirling reinforcing, θ_1_ and θ_2_ are >-3 during each acupuncture stimulus. So synchronous spikes of neurons 1-2 (Figure 5D, blue raster) are not only related to θ_12_ but also to θ_1_ and θ_2_. For synchronous spike events of neurons 1-3 and of neurons 2-3 (Figure 5D, cyan and red raster), first-order spike correlations can be ignored. Second-order spike correlations θ_13_ and θ_23_ are, respectively, their main considerations.

For the lifting-thrusting reducing manipulation, analysis results are shown in Figure 6. Similarly, results are same as twirling reducing, except for the characteristic of volatility. In addition, only θ_1_ among the first-order spike correlations is larger than −3 during each acupuncture stimulus. So first-order spike correlations are not main consideration for synchronous spikes. Second-order spike correlations, respectively, represent corresponding order synchronous spike events.

**Figure 6:** Estimation of spike correlations for acupuncture data evoked by lifting-thrusting reducing. **(A)** Ensemble spike activities. The number of neurons is *N* = 3 and the number of trials is *n* = 20. **(B)** Rates of joint spike: η_12_, η_13_, η_23_, and η_123_. **(C)** First-order spike correlations: θ_1_, θ_2_, and θ_3_ (green, pink, and yellow solid lines). **(D)** Second-order spike correlations: θ_12_, θ_13_, and θ_23_ (blue, cyan, and red solid lines). Raster with different colors at the bottom show the timing of corresponding order synchronous spikes.

## Discussion

This paper introduces the concept of spike correlation and builds a log-linear model to describe ensemble spike activities evoked by four acupuncture manipulations. Then according to the idea of the state-space model, ensemble spike trains are defined as observation variables and spike correlations are defined as unknown state variables, which are estimated by the Bayesian theory. Results show that under the condition of acupuncture reducing manipulations, the third-order spike correlation does not exist. This is the primary reason that synchronous spikes are significantly less in this condition.

In this paper, we judge the existence of the high-order spike correlation by the goodness-of-fit of three hierarchical models and their AICs. Readers can also test the presence of high-order spike correlation by the Bayes factor. The Bayes factor is the ratio of two likelihood functions, which is defined as *BF* = *p*(*y*|*M*_1_)/*p*(*y*|*M*_2_). *M*_1_ represents the model containing the high-order spike correlation. When the value of the Bayes factor is larger than 1, it indicates that the experimental data supports model *M*_1_ and the high-order spike correlation exists.

The article "Spiking Correlation Analysis of Synchronous Spikes Evoked by Acupuncture Mechanical Stimulus" was retracted in 2023. Reasons: plagiarism; overlap with other authors' work.

Acupuncture is a kind of the discrete stimulation. Therefore, the log-linear model is time-dependent and model parameters (spike correlations) are time-varying. Meanwhile our model contains spike correlations of each order and we can estimate the “pure” high-order spike correlation. This makes it possible to discuss the effect of high-order spike correlation on a low-order synchronous spike event. In addition, the correlation analysis in this paper is based on a large number of sample data. The spike event of neurons is a stochastic process. One or two experiments cannot reflect synchronous spike activities of the neural ensemble. Therefore, the result based on a small amount of sample data is unreliable. This is a new view to analyze acupuncture neural electrical signals and will become an important scientific method for the quantitative analysis of the acupuncture response system.

## Data Availability Statement

The datasets for this article are not publicly available because participants did not provide consent to have their data released. Requests to access the datasets should be directed to Jiang Wang, jiangwang@tju.edu.cn.

## Author Contributions

QQ, Y-JL, B-NS, Y-QC, C-XH, Y-MQ, and JW designed and performed the research as well as wrote the paper. All authors contributed to the article and approved the submitted version.

## Conflict of Interest

The authors declare that the research was conducted in the absence of any commercial or financial relationships that could be construed as a potential conflict of interest.
